# Drug Response Prediction Based on 1D Convolutional Neural Network and Attention Mechanism

**DOI:** 10.1155/2022/8671348

**Published:** 2022-09-17

**Authors:** Zhu Mingxun, Meng Zhigang, Wang Jingyi

**Affiliations:** ^1^School of Economics and Management, Changsha Normal University, Changsha, Hunan 410003, China; ^2^School of Computer Engineering and Applied Mathematics, Changsha University, Changsha, Hunan 410003, China; ^3^College of Economics and Trade, Hunan Institute of Biomechatronics Vocational Technology, Changsha 410010, China

## Abstract

There are multiple methods based on gene expression, copy number variation, and methylation biomarkers for screening drug response have been developed. On the other hand, many machine learning algorithms have been applied in recent years to predict drug response, such as neural networks and random forests for the discovery of genomic markers of drug sensitivity for individual drugs in cancer cell lines. In this paper, we propose a drug response prediction algorithm based on 1D convolutional neural networks with attention mechanism and combined with pathway networks, which combines the individual histological data affecting drug response and considers the topological nature of the pathways to find the subpathways highly correlated with drug response and use this as a feature to predict drug response by training using convolutional neural networks. Thus, the output values will represent the probability of occurrence of each of these two categories. In this experiment, using five-fold cross-validation, the identification accuracy reached an average of 84.6%, which is 4.5% higher than the direct random forest approach for drug prediction with an AUC value. This proves that the use of the one-dimensional1D convolutional neural network with attention mechanism to predict the response of low-grade glioma patients and drugs has better prediction results.

## 1. Introduction

Due to the wide genetic heterogeneity of human cancers, many patients with seemingly identical tumor types always perform differently to the same drug therapies [1]. Despite the current efforts to develop cancer therapies, these therapies are usually effective for only some patients, while the rest will miss the optimal time for treatment. One way to address this problem is to identify and apply molecular biomarkers as a way to accurately predict individual responses to anticancer drugs. With the rapid development of high-throughput technologies and the reduction in cost, this has opened the door for researchers to assess the impact of multiple molecular features on drug response and identify reliable biomarkers to further establish valid predictors [2, 3].

In the last decades, there have been many approaches to predict drug response by genomic characterization. There are multiple methods based on gene expression [4], copy number variation (CNV) [5, 6], and methylation [7] biomarkers for screening drug response have been developed. For example, Zhang et al. [8] proposed a method to identify significantly related biomarkers and then used hierarchical sequential logic models to predict drug responses, leading to the development of sequential genomic classifiers. Also He et al. [9] provides a comprehensive review of the clinical relevance of CNV to drug efficacy. There are also several existing data resources such as CancerDR [10], GEAR [11], and CARD [12] that cover many molecular markers associated with drug response. Although these have contributed significantly to preclinical studies, most approaches to identifying biomarkers and predicting drug response assume that major genes act independently, ignoring the functional relationships between genes in biological pathways. Drug response is not determined by a few independent genes, and in fact alterations in signaling pathways largely determine the efficacy of kinase inhibitors used in the clinic [13].

On the other hand, many machine learning algorithms have been applied in recent years to predict drug response, such as neural networks and random forests for the discovery of genomic markers of drug sensitivity for individual drugs in cancer cell lines [14]. Daemen et al. used least squares support vector machines and random forests algorithms to integrate molecular features at various levels of the genome to predict drug response in breast cancer cell lines [15]. Menden et al. used neural networks to predict drug response, where each drug-cell line pair integrated the genomic features of the cell line and used the chemical properties of the drug as a predictor [16] .Cortés-Ciriano et al. modeled chemical and cell line information in machine learning models such as random forest (RF) or support vector regression model to predict the drug sensitivity of numerous compounds screened from the NCI60 panel against 59 cancer cell lines [17]. Although various methods have been developed to computationally predict drug responses in cell lines, many challenges remain in obtaining accurate predictions.

In this paper, we propose a drug response prediction algorithm based on convolutional neural networks and combined with pathway networks, which combines the individual histological data affecting drug response and considers the topological nature of the pathways to find the subpathways highly correlated with drug response and use this as a feature to predict drug response by training using convolutional neural networks. The method first combines multiple histologies of genes and combines the network properties of the pathways to calculate the most relevant subnetworks to drug response, and then uses these subnetworks as feature modules, and uses the degree of expression of genes in these modules on different histologies as training features of the convolutional neural network model for prediction of drug response in different individuals. The algorithm in this paper has low complexity and is able to identify the functional pathway status of genes associated with drug response, and experimental results show that the algorithm is more accurate than traditional machine learning methods.

## 2. Drug Reaction Feature Extraction and Classification

### 2.1. Data Sources

The TCGA database contains multiomics data from many cancer and normal samples as well as drug response data, here we collected expression, methylation, copy number variation, and drug response data from 130 patients with low grade glioma in TCGA.

### 2.2. Methods

The specific process of convolutional neural network-based drug response prediction algorithm: firstly, drug signature genes are identified and scored comprehensively, subpathway screening is performed using simulated annealing algorithm and subpathway multiomics scoring is performed to construct the convolutional neural network model.

#### 2.2.1. Identifying and Scoring Drug Signature Genes

Current studies have shown that drug response is closely related to molecular characteristics such as gene expression, methylation, and copy number. Identifying drug response signature molecules is essential for predicting drug response. Firstly, we dichotomized the drug response profiles of 130 patients in the TCGA database into four categories for drug response profiles, which we dichotomized into two types, i.e. responders (including complete and partial response) and nonresponders (including stable disease and progressive disease). And this label was used as the label for subsequent classification.

For the multidimensional histological data of 130 hypoglioma patients obtained from the TCGA database, we combined the dichotomized labels with the three histological data separately and processed them using the one-way Roger set regression algorithm to identify the drug-sensitive characteristic molecules of each histology and obtain their significance index *p* values as well as coefficient values, respectively.

To integrate the characteristic molecules from multiple histologies, a new composite scoring was constructed, where the *p* values of the significant indicators for each gene in each histology were log processed and summed to yield a composite scoring for the gene. This integrated scoring allows the complementary nature of the histological information to be highlighted, resulting in a more comprehensive presentation of drug-sensitive signature molecules and improved accuracy in the subsequent predictive analysis.

#### 2.2.2. Subpathway Screening and Subpathway Multiomics Scoring Using Simulated Annealing Method

The 130 samples were randomly divided in half into training and test sets, and the training set was scored for gene synthesis, and then this scoring was mapped to the KEGG pathway as the weight of the gene, and then the simulated annealing algorithm was applied to identify the subpathways that were strongly associated with drug sensitivity. In this way, the data from the different three dimensions are integrated and their individual molecular features are expanded into functional modules based on the topology of the network in order to predict individual drug responses comprehensively at the functional level.

The subpathways were then screened for the number of genes contained in the subpathways greater than or equal to 3, and the *p* value of the significance index of the subpathways was required to be less than or equal to 0.05. The screened subpathways were used as features, and the expression values of the genes in the subpathways in each histology were combined to construct the feature scores of the subpathways with respect to each histology.

The scoring on the three histologies of these subpathways are then used as new classification features, and then the convolutional neural network algorithm is applied to train the classifier model.

#### 2.2.3. Construction of Convolutional Neural Network Model

The 130 sample data were divided into a training set and a test set, each with multiple features, each containing (mRNA, Methyl, and CNV).

1. Input data: The data were preprocessed to contain 17 time slices per data record (the data were derived from subpathway screening using simulated annealing method, so each time interval contains 3 kinds of data mRNA, Methyl, and CNV). When performing subpathway screening, the three data mRNA, Methyl, and CNV are stored. This results in a 17 x 3 matrix. As the data needs to be spreading into a vector of length 51 and then passed into the neural network. The first layer of the network must then be deformed into the original 17 x 3 shape
2. The first 1D CNN layer: The first layer defines a filter (also called a feature detector) with a height of 1 (also called the convolutional kernel size). Only when a filter is defined can the neural network learn a single feature in the first layer. This may not be enough, so we will define 100 filters. This way we train 100 different features in the first layer of the network. The output of the first neural network layer is a 17 x 100 matrix. Each column of the output matrix contains the weight of one filter. With the defined kernel size and considering the input matrix length, each filter will contain 17 weight values
3. Maximum value pooling layer: To reduce the complexity of the output and to prevent overfitting of the data, pooling layers are often used after the CNN layer. In this experiment, we chose a pooling layer of size 3. This means that the output matrix of this layer is only one-third the size of the input matrix
4. Dropout layer: The dropout layer randomly assigns zero weights to the neurons in the network. Since a ratio of 0.5 is chosen for this experiment, 50% of the neurons will be zero-weighted. By this operation, the network is less sensitive to small changes in the data. Therefore, it is able to further improve the accuracy of processing invisible data. The output of this layer is still a 1 x 1700 matrix
5. Using dense layer 1: In order to take the features extracted earlier, in dense after a nonlinear change, extract the association between these features and finally map them to the output space, the vector of length 1700 is reduced to a vector of length 512. Also to be able to converge faster
6. Using dense layer 2: The vector of length 512 is reduced to a vector of length 256 for faster convergence and more accurate classification in the subsequent fully connected layer
7. Fully connected layer with Softmax activation: The last layer will reduce the vector of length 256 to a vector of length 2, since we have 2 categories to predict (i.e., “responsive” and “unresponsive”). Softmax is used as the activation function. It forces the sum of all 2 output values of the neural network to be one. Thus, the output values will represent the probability of occurrence of each of these two categories

#### 2.2.4. Adding Attention Mechanism

Adding an attention mechanism to the model in this paper involves three main parts.

(1) calculating the similarity between the input vector and the metric environment vector to find the part that needs attention in the current situation (score-function), (2). calculating the relevant attention weights while using the function normalization (Alignment-function), and (3). obtaining the output vector (Vector function) according to the attention weights. The calculation formula is as follows:

(1) $$\begin{array}{c} e_{\text{i},j}=v_{a}^{T}\tanh\left(W_{a}*c+U_{a}*y_{i}\right),\\ \alpha_{i,j}=\frac{\exp\left(e_{i,j}\right)}{\sum_{k=1}^{T_{z}}\exp\left(e_{i,k}\right)},\\ z_{i}=\underset{i}{\sum }\alpha_{i,j}*y_{i.} \end{array}$$

The structure is as follows (see Figure 1):

## 3. Experimental Results and Analysis

In this experiment, we analyzed the multidimensional histological data and drug response data of 130 low-grade glioma patients in the TCGA database and combined the pathway information to predict the response of brain low-grade glioma patients to temozolomide drug, although high stability was not observed in the five-fold cross-validation process due to the limitation of the number and quality of samples, the current methodological process can basically predict the response of samples in the TCGA database accurately and stably. This methodological process is not limited to cancer and drugs, but can also be applied if there are sufficiently large and good quality data, which provides the potential for the discovery of biomarkers that are currently needed for therapeutic use in the clinic, although the clinical translation of biomarkers is still slow. Some contributions can be made to personalize drug use for cancer patients.

In this experiment, random forest one-dimensional convolutional neural network and one-dimensional convolutional neural network with attention mechanism were used for prediction, respectively. Among them, the 1D convolutional neural network with attention mechanism method used in this paper applied a five-fold cross-validation (see Figures 2–6).

This results in an average accuracy of 84.6% on the test set after doing a five-fold cross-validation, which is 3.5% higher than the direct random forest approach (see Figure 7) for drug prediction with an AUC value.

This proves that the use of one-dimensional convolutional neural network to predict the response of low-grade glioma patients and drugs has better prediction results (see Table 1).

The accuracy results of the three methods are shown in the following Table 1:

## 4. Conclusion and Discussion

The identification accuracy in this experiment utilizing five-fold cross-validation was 84.6 percent, which is 4.5 percent higher than the direct random forest strategy for drug prediction with an AUC value. This shows that using 1D convolutional neural networks with attention mechanism and combined with pathway networks to predict the response of low-grade glioma patients to medicines is more accurate. This methodological process is not limited to cancer and drugs, but can be used in any situation where there is enough large and high-quality data, allowing for the discovery of biomarkers that are currently needed for therapeutic use in the clinic, despite the fact that biomarker clinical translation is still slow. Some contributions can be made to help cancer patients customise their medicine use.

Predicting clinical drug response from molecular data in human cancers is an important goal in precision medicine. This paper combines the response records of patients with low-grade gliomas of the brain to Timozolomide drugs in the TCGA database with their multidimensional histological data to evaluate different molecular data types in predicting clinical drug response in the context of functional modules. We found that the predictive power of multidimensional histology data combined with pathway data was much greater than that of single histology data. This method of constructing characteristic subpathways combines pathway classification features, thus improving the accuracy and stability of prediction.

The next step in the future could be to extend the work to the identification of biomarkers so that the prediction algorithm can not only predict the link between biomolecules and drug response, but also reveal novel biomarkers about cancer therapy.

## Figures and Tables

**Figure 1:** Structure of attention mechanism.

**Figure 2:** First fold cross-validation results.

**Figure 3:** Second fold cross-validation results.

**Figure 4:** Third fold cross-validation results.

**Figure 5:** Fourth fold cross-validation results.

**Figure 6:** Fifth fold cross-validation results.

**Figure 7:** ROC curve of random forest method.

**Table 1:** Comparison results of accuracy rates.

Model name	Recognition accuracy
Random forest	81.1%
One-dimensional convolutional neural network	81.6%
One-dimensional convolutional neural network with attention mechanism added	84.6%

## Data Availability

The data used to support the results of this study are provided by Zhumingxun under license and therefore are not available free of charge. Requests for access to these data should be sent to Dr. Zhu. (zhumingxun@163.com).
